The article "The Clinical Application of Combined Ultrasound, Mammography, and Tumor Markers in Screening Breast Cancer among High-Risk Women" was published in 2022. Journal: Comput Math Methods Med.

# The Clinical Application of Combined Ultrasound, Mammography, and Tumor Markers in Screening Breast Cancer among High-Risk Women

**DOI:** 10.1155/2022/4074628

**Published:** 2022-07-15

**Authors:** Lin Sun, Min Qi, Xiaomei Cui, Qinghua Song

**Affiliations:** ^1^Department of Clinical Laboratory, Yantaishan Hospital, Yantai 264000, China; ^2^Department of Clinical Laboratory, The Second Affiliated Hospital of Shandong University of Traditional Chinese Medicine, Jinan 250001, China; ^3^Department of Obstetrics, Affiliated Qingdao Central Hospital, Qingdao University, Qingdao 266042, China; ^4^Department of Medical Imaging, Qingdao Women and Children's Hospital, Qingdao 266034, China

## Abstract

In order to explore the clinical application value of color Doppler ultrasound (CDUS), mammography (MAM), and serum tumor marker carbohydrate antigen 153 (CA153) in screening breast cancer (BC) for high-risk women, a total of 38,241 women were surveyed by epidemiological questionnaire on BC high-risk factors. A total of 10,821 cases were screened, accounting for 28.30%. They were randomly divided into US, MAM, and CA153 and combined examination group which has no significant difference in high-risk factors. Breast cancer in high-risk population was screened by CDUS, MAM, and CA153 and combined examination. CA153 was detected by electroluminescence method. The positive detection rate of BC was 360.41/100,000 (39/10,821). The overall difference in the positive detection rate of BC among 10,821 cases in all age groups was statistically significant. The sensitivity and negative predictive value of combined examination were significantly improved compared with each single examination. Combined examination for BC screening can significantly improve the sensitivity of BC early diagnosis and reduce the missed diagnosis rate.

## 1. Introduction

With the change of people's lifestyle, living environment, and the increase of living pressure, malignant tumor has become one of the most important diseases endangering the health of Chinese residents. Among them, BC is a common malignant tumor in women. In recent years, its incidence rate is increasing, and the age of onset has gradually become younger, which seriously threatens women's health [1]. The onset of BC is insidious without nonspecific symptoms at early stage, and most of them lost the best opportunity for treatment when they were found in the middle and late stage [2, 3]. The prognosis of BC is closely related to its early detection. Early detection, early diagnosis, and early treatment are not only related to the individual survival effect of BC patients but also become a major issue affecting the national economy and people's livelihood [4]. Therefore, it is particularly important to carry out screening of BC high-risk groups.

At present, the CDUS has become the first choice for the female BC screening which can reveal the internal structure and blood flow of breast masses and observe the morphology, boundary, and internal echo of the lesion and has a strong ability to distinguish solid and cystic masses, but small lesions and calcified lesions easily missed diagnosis and misdiagnose [5, 6]. MAM can image the entire breast with a strong sense of integrity and not easy to miss diagnosis, but with a low resolution for tissue density and inability to clearly show the lesions for dense breast lesions, resulting in low sensitivity and specificity for diagnosis [7, 8]. Thus, there are certain limitations in their application alone. In this study, three methods including CDUS, AMA, and tumor markers were selected to screen BC in high-risk women. Compare the difference between the value of the combined examination and each single examination to provide a basis for better screening of BC in high-risk groups.

## 2. Research Objects and Methods

### 2.1. Research Objects

From January 2016 to December 2018, a total of 38,241 women aged 30-70 from 31 communities in our city were selected for screening BC at high risk. CDUS, MAM, and serum tumor marker CA153 single and combined examination methods were used for BC screening.

### 2.2. High-Risk Population Screening

Community health service centers publicize the significance and importance of carrying out BC screening to residents through free community diagnosis in communities, distributing of brochures, and household publicity. A questionnaire survey was conducted among female residents aged 30-70 years old who voluntarily participated and sign the informed consent form. Based on the “Harvard Cancer Risk Index” [9], a comprehensive assessment system of individual cancer risk suitable for Chinese population was developed through multidisciplinary expert group discussion and consensus. The respondents completed the “Breast Cancer Risk Assessment Questionnaire” by themselves under the guidance or after being questioned by professionally trained investigators. The basic information of the questionnaire included menarche age, menopause age, delivery history, lactation history, family history of BC, history of benign and malignant breast diseases, dietary habits, changes in postmenopausal weight, and history of long-term use of exogenous estrogen. Each factor has a risk score, and the sum scores of all risk factors constitute the risk score. The risk assessment is performed by collecting the filled data information. Risk scores above 30 were considered high-risk groups and participated in this study.

### 2.3. CDUS Examination and the Criteria

The diagnostic instrument is PHILIPS iU22, and the frequency of the probe is 5-12 MHz. During the inspection, the examinee was asked to take a supine position, raise arms, and place hands behind the head to fully expose the bilateral breasts, supraclavicular fossa, and bilateral axillary areas. Each quadrant of the breast, the supraclavicular fossa, and bilateral axillary regions were scanned. Firstly, the lesion location, morphology, mass size, borders, whether the internal echo is uniform, whether there is attenuation of posterior echo, calcification, and association with surrounding tissues, whether lymph nodes metastasize in axillary and clavicle, and other acoustic images were observed, and then, the shape and distribution of blood flow signals inside and around the lesion were observed, and hemodynamic parameters was also measured [10].

Two-dimensional US images revealed obvious masses which were irregular in shape, blurred in boundary, lobulated, burr-shaped, uneven internal echo and attenuation of the rear echo, and calcification (Figure 1(a)). CDUS showed more abundant blood flow in and around the mass (Figure 1(b)).

### 2.4. Mammography Examination and the Criteria

MAM was performed by a diagnostic instrument GE Senographe 2000D digital MAM machine. In general, internal and external oblique (MLO) and axial (CC) positions were used for photography, and magnification photography or compression photography with small compressors was used for small lesions. The X-ray differential diagnosis of benign and malignant breast diseases is mainly performed from the density, morphology, and indirect signs of the mass. The diagnostic criteria refer to the BI-RADS classification standard (Breast Imaging Reporting and Data System of the American College of Radiology) [11].

MAM examination showed the presence of masses or nodules with irregular, blurred borders, lobular and burr-like changes, micro, granular, or cast calcifications, localized dense infiltration, or skin changes (Figure 2).

### 2.5. Detection of Serum Tumor Marker CA153

Serum tumor marker CA153 was detected by ELecsys-2010 (Roche, Suisse) using electroluminescence method. All operations were carried out strictly according to the operating instructions, and the quality control met the requirements. The normal reference values of tumor markers is CAl53 ≤ 25.00 U/ml. Serum CA153 > 25.00 U/ml was diagnosed as positive.

### 2.6. The Criteria for Combined Examination

In the combined examination, one or more of the positives were judged as positive, and all were negative to judge to be negative.

### 2.7. Statistical Analysis

The data were processed by SPSS 25.0 statistical software. Data were expressed as mean ± standard deviation(^−^*x* ± sd). The comparison of means between groups was performed by analysis of variance, and the comparison of count data was performed by the *χ*^2^ test. *P* < 0.05 was statistically significant.

## 3. Results

### 3.1. Screening Results for High-Risk BC Populations

A questionnaire survey of BC risk factors and assessment of high-risk groups were conducted on 38,241 women. A total of 10,821 eligible people were screened, accounting for 28.30% (10,821/38,241) with an average age of 52.34 ± 10.21 years. They were randomly divided into US group (2705 cases), MAM group (2707 cases), CA153 group (2703 cases), and combined examination group (2706 cases). There was no statistically significant difference in BC risk factors and comprehensive risk scores among the four groups (Table 1), and they were comparable.

### 3.2. Comparison of Positive Detection Rates of BC in High-Risk Groups of All Age

With pathological examination as the gold standard, 39 cases of BC were confirmed by pathology in 10,821 cases with the high-risk group. The positive detection rates of the groups aged 30-39, 40-49, and 50-70 were 152.13/100,000 (3/1972), 539.08/100,000 (24/4452), and 272.91/100,000 (12/4397), respectively (Table 2). The overall difference in the positive detection rate of BC among 10,821 cases in the high-risk group in all age was statistically significant (*χ*^2^ = 7.277, *P* = 0.026) (Table 2). There was a significant difference in the positive detection rate of BC between 40-49 and 30-39 years old (*χ*^2^ = 4.889, *P* = 0.027) and between 40-49 and 50-70 years old (*χ*^2^ = 3.868, *P* = 0.049), but there was no significant difference between the ages of 30-39 and 50-70 years (*χ*^2^ = 0.845, *P* = 0.358) (Table 2).

### 3.3. Comparison of the Value of CDUS, MAM, and CA153 and Combined Examination in Screening BC among High-Risk Population

A total of 426 of the 10,821 cases were confirmed by pathology, including 39 cases of BC and 387 cases of benign lesions. The results of CDUS, MAM, and CA153 and combined examination were determined to be true positive or true negative if they were consistent with pathological diagnosis, otherwise as false positive or false negative. Compared with each single examination, the sensitivity and negative predictive value of the combined examination were significantly improved (Table 3).

## 4. Discussion

The pathogenesis of BC is not completely clear. It is currently believed that the occurrence of BC is associated with menarche history, menopause history, long-term use of exogenous estrogen history, menstrual marriage history, BC family history, etc. [12, 13]. Aiming at the high-risk factors of BC, screening high-risk BC populations has great significance for the early diagnosis and early clinical intervention of BC. BC screening includes self-examination, clinician physical examination, imaging examination, and serum tumor marker examination. Imaging examinations mainly include breast CDUS, MAM, and magnetic resonance imaging (MRI). Imaging examination has been proved to be effective in improving the early diagnosis of BC [14]. MRI is not suitable for BC screening because of its complicated operation and high cost; thus, US and MAM are more suitable for BC screening [15]. In addition, serum tumor marker detection which is an in vitro diagnostic test with the advantages of noninvasive, nonrisk, simple operation, and low cost is often used for BC screening.

The advantages of CDUS are noninvasive, nonrisk, convenient, and free of radiation. It can be suitable for any age, whether pregnant, lactating women, or the elderly, and can be repeated. The patient has good compliance. It has been widely used in clinical BC screening. US can scan the lesion from multiple angles and directions to clearly show the characteristics of the lesion, including position, size, shape, boundary, internal echo, and calcification, and clearly display surrounding tissue of the lesion area to judge the invasion of the surrounding tissue [16]. At the same time, according to the characteristics of tumor angiogenesis and blood flow around the lesion, the direction, velocity, and state of blood flow can be analyzed to clearly reflect the information of bleeding flow dynamics and further identify benign or malignant breast mass [17]. US can effectively distinguish cystic lesions from solid lesions [18] and has a strong diagnostic ability for invasive ductal carcinoma, especially for dense breast lesions [19]. The disadvantage of US is that the diagnostic level of the US physician has a large artificial influence on the diagnosis result, it is difficult to find some microcalcification foci and small lesions with unclear echo, and the missed detection rate of ductal carcinoma in situ is high [20, 21].

MAM is also one of the main methods of BC screening. The advantage is that the entire breast can be imaged, the overall sense is strong, and it is not easy to miss the diagnosis. Smaller lesions, calcification of the lesions (especially microcalcifications), and glitches are clearly shown. It has extremely high clinical diagnostic value for ductal carcinoma in situ which is easy to be missed by US, effectively reducing never diagnosis and misdiagnosis. In addition, the MAM examination can transmit the image data in digital form to meet the needs of remote consultation. It is an irreplaceable examination method for BC screening, especially for the diagnosis of tumors with malignant calcification. The disadvantages are that the resolution of tissue density is low and the lesions of dense breast lesions cannot be clearly displayed [7, 8]. Moreover, it is insufficient for the identification of cystic mass and solid mass and the diagnosis of invasive ductal carcinoma. In addition, this test has a large radiation dose and is not suitable for pregnant women, lactating women, and repeated inspections.

Tumor markers are a class of substances secreted by tumor cells or produced by the interaction between tumor and host during the carcinogenesis of tissue cells, including some glycoproteins, hormones, enzymes, and other substances, which can be detected in tissues or peripheral body fluids [22]. Serum tumor markers have gradually become an important means of BC screening, and detecting the level of relevant tumor markers is conducive to the early screening of BC [23]. CA153 is a kind of high molecular weight glycoprotein, which exists in the cell membrane of breast tissue [22]. The cytoskeleton is destroyed when cells become cancerous, resulting in the cell surface antigens falling off and being released into the blood and the increased content of CA153 levels in peripheral blood [24]. CA153, as a classic tumor marker for the diagnosis of BC, has become a routine examination item for women's health examination. However, the sensitivity and specificity of serum CA153 alone as a screening program for BC high-risk population are obviously insufficient.

If BC screening is performed for all females of appropriate age, both the cost and workload are huge and impractical. Therefore, it is necessary to screen out the high-risk population for BC screening on the basis of the high-risk factors of BC. In this study, 38,241 aged 30-70 women were screened for BC risk factors, and a total of 10,821 cases were screened. CDUS, MAM, and serum CA153 were used for single or combined examinations. With pathological diagnosis as the gold standard, a total of 39 cases of BC were screened out, including 15 cases of early stage (stage 0 and stage I), which could be completely cured by early surgery, so the screening effect was significant. Each single examination has its own advantages and disadvantages. The positive detection rate and negative predictive value of the combined examination were significantly higher than those of single examination.

US examination has better resolution of soft tissues, while MAM has a low resolution of tissue density, especially the inability to clearly show dense breast lesions which can easily cause missed diagnosis [25]. Younger women have higher breast tissue density, and US is better than MAM examination, while older people have the opposite [26, 27]. At the same time, the detection of MAM for lesion calcification and carcinoma in situ is better than US, while US has a high detection rate for invasive ductal carcinoma, suggesting that the combined examination of the two is obviously complementary [28]. In addition, the tumor marker CA153 shows an increasing trend in peripheral blood when some BC imaging manifestations are not typical. Therefore, it is a good supplementary experiment for imaging examinations, although this study showed that serum CA153 is not sensitive for screening BC in high-risk populations (44.44%), which is related to early screening. CA153 has not been released into the blood to cause false negatives in early BC. Thus, CA153 is still an essential screening item for BC screening. This study also showed that women aged 40-49 has a high incidence of BC, suggesting that regular medical examinations should be performed to achieve early detection and early treatment.

## 5. Conclusion

With the increasing incidence of BC, it is necessary to explore its screening model. By screening high-risk groups, early BC can be detected, which can significantly improve the clinical cure rate. US, MAM, and CA153 are commonly used screening methods, but the value of a single examination is limited. The combined test can complement and confirm each other, thereby reducing misdiagnosis and maximizing the positive detection rate of BC screening.

## Figures and Tables

**Figure 1:** CDUS images of BC. (a) Two-dimensional US images. The arrow showed a two-dimensional US image showing a single nodule in the left breast, about 0.77 × 0.54 cm in size, with irregular shapes, fuzzy nodule edges, visible burrs, uneven internal echo, low echo, and spotting echo. (b) Color Doppler flow image. Arrows indicated abundant blood flow signals around the nodule. Color Doppler diagnosis was B1-RADS 5.

**Figure 2:** MAM image of BC. (a) Axle position (CC). (b) Internal and external oblique position (MLO). The arrow showed a nodule lower-inner of the left breast with a size of about 2.2 × 2.1 cm, unclear edge, lobular sign, and elongated burr-like changes. MAM diagnosis was B1-RADS 5.

**Table 1:** Comparison of the distribution of high-risk factors among four groups of high-risk BC populations.

Factors	US group (*n* = 2705)	MAM group (*n* = 2707)	CA153 group (*n* = 2703)	Combined detection group (*n* = 2706)	*χ* ^2^/*F*	*P*
Age (years)					3.285	0.772
30-39	485	502	495	490		
40-49	1149	1096	1112	1095		
50-70	1071	1109	1096	1121		
Menarche age (years)					3.984	0.263
<12	336	295	317	298		
≥12	2369	2412	2386	2408		
Menopausal status					1.691	0.639
Premenopausal	2060	2094	2069	2056		
Postmenopausal	645	613	634	650		
Family history of BC					0.792	0.851
Yes	180	165	175	170		
No	2525	2542	2528	2536		
Breast disease history					1.538	0.674
Yes	157	137	145	150		
No	2548	2570	2558	2556		
Long-term use of exogenous estrogens					2.962	0.397
Yes	39	50	41	35		
No	2666	2657	2662	2671		
Delivery history					2.002	0.572
Yes	2545	2562	2561	2568		
No	160	145	142	138		
Obesity					1.210	0.751
Yes	262	252	240	257		
No	2443	2455	2463	2449		
Risk score (^−^*x* ± *s*)	39.23 ± 6.59	37.67 ± 7.12	38.56 ± 6.57	39.12 ± 7.01	0.882	0.769

**Table 2:** Comparison of positive detection rates of BC in high-risk groups of all age.

Group	Pathology		*χ* ^2^	*P*
	Positive (*n*)	Negative (*n*)		
30-39 years (*n* = 1972)	3	1969	4.889	0.027
40-49 years (*n* = 4452)	24	4428	3.868	0.049
50-70 years (*n* = 4397)	12	4385	0.845	0.358
*χ* ^2^	7.277			
*P*	0.026			

**Table 3:** Comparison of the value of CDUS, MAM, and CA153 and combined examination in screening BC among high-risk population (%).

Detection indicator	Sensitivity	Specificity	Accuracy	Positive predictive value	Negative predictive value
US	70.00	91.51	88.10	60.86	94.17
MAM	66.67	90.63	86.84	57.14	93.55
CA153	44.44	89.61	81.05	50.00	87.34
Combined examination	90.91^a^	91.67	91.53	68.97	98.02^a^
*χ* ^2^	10.106	0.288	5.548	1.710	8.537
*P*	0.018	0.962	0.136	0.635	0.036

^a^Compared with each single examination, *P* < 0.05.

## Data Availability

The datasets used and/or analyzed during the present study are available from the corresponding author on reasonable request.
